The article "Genipin suppression of growth and metastasis in hepatocellular carcinoma through blocking activation of STAT-3" was retracted in 2022. Reasons: plagiarized images; unreliable results or conclusions.

# Genipin suppression of growth and metastasis in hepatocellular carcinoma through blocking activation of STAT-3

**DOI:** 10.1186/s13046-020-01654-3

**Published:** 2020-08-02

**Authors:** Ming Hong, Selena Lee, Jacob Clayton, Wildman Yake, Jinke Li

**Affiliations:** 1 Science and Technology Innovation Center, Guangzhou University of Chinese Medicine, Guangzhou, China; 2 Institute of Clinical Pharmacology, Guangzhou University of Chinese Medicine, Guangzhou, China; 3 Department of Pharmacology & Toxicology, University of Kansas, Lawrence, KS USA

## Abstract

**Background:**

The signal transducer and activator of transcription-3 (STAT-3) can facilitate cancer progression and metastasis by being constitutively active via various signaling. Abundant evidence has indicated that STAT-3 may be a promising molecular target for cancer treatment.

**Methods:**

In this study, a dual-luciferase assay-based screening of 537 compounds for STAT-3 inhibitors of hepatocellular carcinoma (HCC) cells was conducted, leading to the identification of genipin. Effects of genipin on HCC were assessed in a patient-derived xenograft nude mice model. Western blotting assay, chromatin immunoprecipitation (ChIP) assay, molecular docking study, tube formation assay, three-dimensional top culture assay, histological examination, and immunofluorescence were utilized to evaluate the regulatory signaling pathway.

**Results:**

Our research demonstrated that genipin suppresses STAT-3 phosphorylation and nuclear translocation, which may be attributed to the binding capacity of this compound to the Src homology-2 (SH2) domain of STAT-3. In addition, the therapeutic effects of genipin in a patient-derived HCC xenograft nude mice model were also demonstrated.

**Conclusions:**

In conclusion, genipin showed therapeutic potential for HCC treatment by interacting with the SH2-STAT-3 domain and suppressing the activity of STAT-3. In the future, further research is planned to explore the potential role of genipin in combination with chemotherapy or radiotherapy for HCC.

## Background

The signal transducer and activator of transcription-3 (STAT-3) was originally identified as a critical mediator of the IL-6-type cytokine signal pathway and described as an acute phase response factor (APRF) [1, 2], which can operate as a transcription factor of various cytokines, interferons, hormones, and growth factors [3]. After dimerization, STAT-3 can transfer to the nucleus and act as a transcription activator. Phosphorylation of tyrosine 705 residue induced by epidermal growth factor (EGF) or interleukins can activate STAT-3 in cells [4]. STAT-3 can facilitate cancer progression and metastasis by being constitutively active via various signaling, as previously described [5, 6]. Abundant evidence indicates that STAT-3 may be a promising molecular target for cancer treatment. Inhibiting of STAT-3 activity can be divided into two categories: regulating upstream genes of STAT-3 or directly binding to STAT-3 and suppressing its activity [7]. Although the direct targeting of STAT-3 is extremely difficult, novel targeting agents continuously emerge. For example, Bai et al. recently found a highly selective small-molecule degrader of STAT-3, i.e., SD-36, which could suppress lymphoma cell growth and inhibit tumor progression in a mice model. In addition, several natural products, such as alantolactone and osthole, can suppress the phosphorylation and activation of STAT-3 as well as inhibit tumor progression in breast cancer by directly binding with the SH2 domain of STAT-3 [8, 9]. However, none of these candidate agents have been assessed for their binding affinity to STAT-3. Their selectivity with STAT-3 and other STAT family proteins still needs further exploration.

Hepatocellular carcinoma (HCC) is a highly fatal malignant disease that is the third leading cause of cancer-related deaths in developing countries [10]. Most HCC patients are diagnosed at an advanced stage, and therefore these patients have few chances for radical therapy. Although major progress in HCC treatment has been achieved in recent years, HCC patients still have a poor prognosis, with high rates of metastasis and post-operative recurrence [11]. Thus, further exploring the underlying molecular mechanisms of HCC and developing highly effective therapies for HCC are urgently needed. Persistent activation of STAT-3 has been found in the majority of HCC patient tissues instead of para-carcinoma tissue and has been closely associated with poor prognosis [12]. Studies have increasingly shown that STAT-3 plays critical roles in HCC growth and metastasis. Therefore, STAT-3 may be a promising therapeutic target in HCC treatment. Clinical studies have explored the potential benefits of STAT-3-targeted agents used either alone or in combination with chemotherapy in HCC patients. Some of these agents have revealed a promising clinical efficacy and safety profile in clinical trials [13].

In this study, a dual-luciferase assay-based screening of 537 compounds for STAT-3 inhibitors was conducted, leading to the identification of genipin. Further research demonstrated that genipin suppresses STAT-3 phosphorylation and nuclear translocation, which may be attributed to the binding capacity of this compound to the SH2 domain of STAT-3. Furthermore, the therapeutic effects of genipin were also evaluated in a patient-derived HCC xenograft mice model.

## Materials and methods

### Cell lines

MHCC97L, HepG2, and LO2 cells were obtained from the American Type Culture Collection (Manassas, VA). The cells were cultured in RPMI 1640 medium containing 10% FBS at 37 °C in a humidified atmosphere containing 4% CO_2_. Media were supplemented with antibiotics including 150 μg/ml of streptomycin and 50 U/ml of penicillin.

### Luciferase reporter assay

The luciferase reporter system was applied using the pGMSTAT-3-Luc plasmid for detecting the activation of STAT-3. The plasmid was purchased from Genomeditech (#GM-021003, Shanghai, PRC) and transfected into cells following the instructions from a previous study [14]. Before plasmid transfection, MHCC97L cells were cultured in a 12-well plate for 12 h. Co-transfection of pRL-SV40 (Renilla luciferase) and pGMSTAT-3-Luc was conducted by Lipofectamine 3000 (Thermo Scientific, USA) in MHCC97L cells. One day after transfection, MHCC97L cells were exposed to the test chemicals from our internal chemicals library, which were provided by Prof. Ma of the Xi’an Jiao Tong University Medical School for 12 h [15]. The exposure time and concentration of the chemicals library were referred to previous studies [15]. Geniposide was purchased from Sigma Co. Ltd. (purity> 99% by HPLC). The luciferase signal was analyzed using the dual-luciferase reporter systems as previously described [16]. The activation of STAT-3 regulated by candidate agents was analyzed by the proportion between the value of Renilla and firefly luciferase activity.

### Immunoblotting

Immunoblotting assay was conducted as previously described [17]. The nuclear and cytosol proteins were extracted using the Nuclear Protein Extraction kit (Fermentas, USA). The related primary antibodies and secondary antibodies were purchased from Abcam (Cambridge, USA). The following primary antibodies were used for immunoblots at the appropriate dilutions: p-stat3-Tyr705 (1:1000), p-stat3-Ser727 (1:1000), stat3 (1:1000), GAPDH (1:5000), Surviving (1:500), Mcl-1 (1:1000), Bcl-2 (1:1000), VEGF (1:500), MMP2 (1:1000), Socs3 (1:500), PARP (1:500), Cleavage PARP (1:500), N-cadherin (1:1000), E-cadherin (1:1000), Vinmentin (1:1000), and Fibronection (1:500).

### Real-time PCR

Total RNA was isolated using TRIzol (Sigma, USA) following the instructions of the manufacturer. The purified RNA was then reverse-transcribed to cDNA with the Invitrogen SuperScript IV kit. Real-time PCR experiments were conducted using the SYBR Green PCR Kit (QIAGEN, China) and reactions were performed for 40 cycles in standard mode using the Bio-Rad CFX96 PCR System. The primers used in this study are shown in Supplementary Table 3. Each reaction was performed in triplicate.

### Cell viability assay

Cell viability was examined by using the 3-(4,5-dimethylthiazol-2-yl)-5-(3-carboxymethoxyphenyl)-2-(4-sulfophenyl)-2H-tetrazolium (MTS) assay as previously described [3]. Absorbance was recorded at 490 nm using a Bio-rad PR-4100 microplate reader (Hercules, USA). Each reaction was performed in triplicate.

### Immunofluorescent staining

Immunofluorescence staining was performed referred to previous studies [18]. Briefly, after fixation with 4% paraformaldehyde, cells were blocked and hybridized with the indicated primary antibodies for 12 h. Next, fluorescein isothiocyanate (FITC)-conjugated secondary antibodies were added and incubated for 2 h; 4′,6-diamidino-2-phenylindole (DAPI) was used for nuclear staining. The fluorescent expressions of the target marker and nucleus were visualized by a confocal microscope (Olympus, Japan).

### Electrophoretic mobility shift assay

Electrophoretic mobility shift assay (EMSA) was conducted to evaluate the DNA-binding activity of STAT-3 in genipin-treated HCC cells. In brief, following transfection of HCC cells for 72 h, nuclear proteins from each sample were extracted with a Nuclear Extraction kit (Sigma, USA) and subjected to EMSA following the manufacturer’s standard protocol using the LightShift® Chemiluminescent EMSA kit (Thermo Fisher Scientific, USA). The STAT-3 target probe was synthesized with a 3′-biotin modification (Invitrogen, USA) and the sequence was 5′-ACG AAC CAT TACGCTCGA CAG CCG-3′, in which the binding region is underlined. EMSA was conducted with STAT-3 EMSA Kit (Thermo Fisher Scientific, USA) following the manufacturer’s instructions. STAT-3 oligonucleotides with infrared dye-labels were as follows: 5′-CTACGGACGTACGAACTGCACGGC-3′ and 3′-ACCTGGACTAACGTCAGCCGCG-5′.

### Chromatin immunoprecipitation assay

HCC cells were added into formaldehyde for immobilizing the protein-DNA complex for chromatin immunoprecipitation (ChIP) assay. Then, cell lysis solution was added. DNA fragments were broken by ultrasound. The related antibodies and beads were added to precipitate the protein-DNA complex. The protein-DNA complex was immunoprecipitated with STAT-3 antibody. Protein A/G agarose beads were applied to incubate with the immunoprecipitate. Next, the samples were washed by PBS and the chromatin-protein complex was reversed. Phenol-chloroform was used to purify the DNA. Then, DNA sequences were validated by qPCR assay. The primers used in ChIP assay were specific for STAT3-binding sites in the promoters of VEGF, SOCS3, and BCL-2.

### Molecular docking study

The three-dimensional (3D) structures of STAT-3 were obtained from the RSCB Protein Data Bank (http://www.pdb.org/) (PDB code: 6NJS) and prepared with Sybyl-X 2.0 (Tripos, St. Louis, MO, USA) for the docking studies [19]. An energy-minimized 3D structure of Genipin (PubChem: 442424) was optimized from NCBI-PubChem (https://pubchem.ncbi.nlm.nih.gov/). The elaborate docking method and reliability validated assay were recorded in the protocol of the Surflex-Dock module of Sybyl-X [20].

### Surface-plasmon-resonance assay

Surface-plasmon-resonance (SPR) assay was applied to further validate the binding affinity of genipin with STAT-3-SH2 protein. The STAT-3-SH2 peptide sequence, FISKERERAILSTKPPGTFLLRFSESSK, was provided by Peptide 2.0 (Fairfax, VA) at > 95% purity. SPR binding assay was performed with Biocore T300 biosensor systems (General Electric, USA) as previously described [21]. All the SPR-based materials were obtained from General Electric Co. The related target proteins were acquired from R&D systems (Minneapolis, USA). Biocore trace was baseline-subtracted and the signals were presented in sensorgrams and determined in RU. Empirically, in the BIOcore technology, 2 ng of analyte bound at the surface gave a response of 1× 10^3^ RU. Equilibrium constants (KD) were calculated with the “affinity” model in Biocore T300 evaluation software version 3.2.

### Tube formation assay

HCC cells were plated in a six-well plate to 95% confluence after 36 h, and then the cells were washed with PBS and the medium substituted by serum-free medium with different concentrations of genipin (0, 10, and 20 μM). Conditioned media were collected after centrifugation at 1200 rpm for 10 min. A total of 2 × 10^4^ HUVECs were seeded into each well of a 12-well plate coated with 200 μL of Matrigel (Sigma, USA), and cultured for 8 h in conditioned medium. Images were captured by an Olympus CKX41 inverted microscope (magnification 100×; Olympus Corp., USA), and analyzed for the extent of tube formation by measuring the tube length and counting the number of tube nodes using ImageJ softwareEach reaction was performed in triplicate.

### Immunohistochemistry assay

Immunohistochemical staining was performed according to previous studies [22]. Antibodies for p-STAT-3 (dilution 1:200) and CD31 (dilution 1:200) were provided by Invitrogen (Carlsbad, CA, USA). Immunohistochemistry assay was performed in an automated system using the Ventana® BenchMark Ultra following the manufacturer’s protocols. The immunohistochemistry slides were examined by three independent researchers. Positivity for p-STAT-3 and CD31 was defined as unequivocally nuclear and cytoplasmic staining of at least 75% of the cancer cells.

### 3D top culture assay

Growth-factor-reduced Matrigel was thawed at 4 °C for 12 h. Matrigel solution (60 μL/well) was added into 24-well plates at 35 °C for 20 min. A total of 2 × 10^5^ MHCC97L cells were re-suspended in 150 μL of serum-free medium and cultured on solidified Matrigel. At 15 min post-cell-attachment, 150 μL of serum-free media with 15% Matrigel and indicated concentrations of genipin were added on top of the plated culture. All experiments were repeated by three independent researchers.

### Animal studies

For details of the construction of HCC xenograft nude mice models, BALB/C mice (4 weeks old, female) were orthotopically implanted with 2 × 10^5^ MHCC97L cells, the reader is referred to our previous studies [19]. The mice were anesthetized by intramuscular injection of 0.2 ml of a solution of 25 mg/kg ketamine and 15 mg/kg xylazine. Two weeks later, the BALB/C mice were randomly divided into a DMSO group (*n* = 8), 25-mg/kg/d genipin treatment group (*n* = 8), and 50-mg/kg/d genipin treatment group (*n* = 8) by i.p. injection. Thirty-five days after treatment, the mice were sacrificed and dissected. The liver tumor weight and lung metastasis nodules were measured by three independent researchers. All animal studies were approved and under the strict supervision of the University of Kansas Committee of Experimental Animal Ethics (Approval No. CF201900239).

For the patient-derived xenograft (PDX) model, HCC cells were collected for constructing a xenograft model as previously described [10]. Seven surgical liver samples were obtained from HCC patients in the Department of Hepatobiliary Surgery of the First Affiliated Hospital of Guangzhou University of Chinese Medicine (Supplementary Table 1). The tumor tissue was incised into small pieces (0.3 cm^3^). Ethanol (75%) was used for surgical disinfection. For anesthesia of the mice, 0.6% lidocaine was applied. For establishing the F1 generation, one piece of the human HCC tissue was sent into the subcutaneous area. When the tumor volume grew to 1 cm^3^, the tumor was dissected into two pieces. One piece of tumor was fixed in 4% formaldehyde solution and the other was further incised into small pieces (0.3 cm^3^). Eight BALB/C mice were transplanted with tumor tissue as described above (F2 generation). The PDX mice model of F3 generation was also conducted as described above. Then, the mice were randomly divided into a DMSO group (*n* = 8), 25-mg/kg/d genipin treatment group (*n* = 8), and 50-mg/kg/day genipin treatment group (*n* = 8) by i.p. injection. Tumor volumes were measured at the indicated time points. All procedures and protocols were approved by the Ethical Committee of the First Affiliated Hospital of Guangzhou University of Chinese Medicine.

### Statistical analysis

All data were presented as mean ± standard deviation (SD) of three independent experiments. The statistical analyses were evaluated by GraphPad Prism using Student’s t-test for comparing two means. Analysis of variance (ANOVA) followed by Tukey’s post hoc test was applied for the statistical analysis when more than two means were compared. *P* values of less than 0.05 were considered statistically significant.

## Results

### Genipin can inhibit the phosphorylation of STAT-3 (Tyr) and decrease the expression of STAT-3 target gene in HCC cells

As a transcription factor, STAT-3 can regulate cell proliferation and angiogenesis through modulation of its downstream target genes, such as Bcl-2, VEGF, and SOCS-3 [23]. To screen novel STAT-3 inhibitory agents, the STAT-3 luciferase reporter system was applied to screen target agents from our internal chemicals library (Fig. 1a, upper panel). After screening 537 compounds, genipin was eventually identified as a novel natural agent for inhibiting the STAT-3 signal pathway. Genipin exhibited significant STAT-3 suppressive activity in MHCC97L and HepG2 cells (Fig. 1a, lower panel). While phosphorylated Y705 has been widely acknowledged to be essential for STAT-3’s transcriptional activity, the function of phosphorylated S727 is still controversial, as this modification has been reported to have both up- and down-regulatory effects on STAT3’s transcriptional activity. Thus, for validating the STAT-3 suppressive effects, p-STAT-3 (Y705) and p-STAT-3 (S727) expression were examined by western blot after genipin treatment. Our results showed that genipin (20 μM) remarkably inhibited the activation of pSTAT-3 (Y705), but failed to affect the protein expression of STAT-3 and p-STAT-3 (S727) (Fig. 1b). In addition, one of genipin’s relative compounds, geniposide, was chosen as a control to confirm the specificity effect of genipin on STAT-3 inhibition. However, our results showed that geniposide has no effect on STAT-3 inhibition in HCC cells (Figs. 1a and b). Cytoplasmic STAT-3 exported to the nucleus is a critical step for regulating its down-stream gene expression. Both immunofluorescent staining and western blotting results confirmed that genipin inhibited nuclear translocation of STAT-3 after being stimulated by Interleukin-6 (IL-6) (Fig. 1c). Furthermore, STAT-3 DNA-binding ability was inhibited by genipin treatment according to the electrophoretic mobility shift assay results (Fig. 1d). Protein tyrosine phosphatases (PTPases) are a group of enzymes that are able to eliminate the DNA binding of STAT-3 [24]; thus, it was our intention to explore whether genipin could inhibit STAT-3 by PTPases in HCC. PTEN, SHP1, and SHP2 are key regulatory PTPases in STAT-3 signal transduction pathways [25]; however, the protein expression of these PTPases has no obvious changes after genipin treatment (Supplementary Fig. 1a). In addition, to further confirm whether genipin inhibits STAT-3 specifically, the activities of STAT-5, STAT-1, STAT-2, mTOR, and MAPK signal pathways were also evaluated by western blotting. Our results indicated that genipin failed to affect the phosphorylation of STAT-5, STAT-1, and STAT-2 as well as the expression of the related proteins in mTOR and MAPK signal pathways (Supplementary Figs. 1b and c). Up to now, it could be concluded that genipin suppressed STAT-3 phosphorylation and nuclear translocation as well as inhibited its DNA-binding ability. STAT-3 dimers exported to the nucleus can activate the promoter of STAT-3 target genes and up-regulate the protein expression of these tumor-related genes, such as Survivin, Bcl-2, MMPs, SOCS3, and VEGF [18]. Western blot assay results further confirmed that genipin treatment decreased the expression of STAT-3 target genes in HCC cells (Fig. 1e). In addition, chromatin immunoprecipitation assay indicated that genipin inhibited the binding affinity of STAT-3 with Bcl-2, SOCS3, and VEGF (Fig. 1f). In summary, the above data revealed that genipin could inhibit STAT-3 phosphorylation (Y705) and suppress its target gene expression in liver cancer.

**Fig. 1:** Genipin suppresses STAT-3 activity in HCC. (**a**) HCC cells were treated with genipin or geniposide for 24 h before transfection with plasmid containing the luciferase reporter gene. Relative luciferase activity was detected using dual-luciferase reporter systems. (**b**) Liver cancer cells were treated with genipin or geniposide for 24 h, and western blot was performed to detect the protein expressions of STAT-3, p-STAT-3 (Y705), and p-STAT-3 (S727). (**c**) MHCC97L cells were seeded in coverslips coated with gelatin, and then genipin (0–20 μM) was added into each sample for 12 h and co-cultured with or without 10-ng/μl IL-6 for 20 min. STAT-3 expression and location was examined by immunofluorescent staining. Cell nuclei were detected by DAPI stanning (left). MHCC97L cells were seeded in coverslips coated with gelatin, and then cells were treated with genipin for 12 h and co-cultured with or without 10-ng/μl IL-6 for 20 min. Cytoplasmic and nuclear STAT-3 levels were detected by western blotting assay (right). (**d**) MHCC97L cells were exposed to genipin for 24 h. STAT-3 DNA-binding activity was analyzed by EMSA assay. (**e**) MHCC97L cells were exposed to genipin for 24 h. The protein expression of STAT-3 target genes were examined by western blot assay. (**f**) MHCC97L cells were exposed to genipin for 24 h. Binding ability of STAT-3 with its target genes was analyzed by ChIP assay. Data presented as mean ± SD. *P < 0.05 and **P < 0.01

### Genipin binds to SH2 domain in STAT-3

Next, whether genipin could directly interact with STAT-3 by in silico assay was explored. As shown in Fig. 2a, genipin was docked nicely into the SH2 domain of STAT-3 (PDB Id: 1GB1). PHE716, LYS626, GLN635, SER636, GLU638, ARG609, LYS591, VAL637, PRO639, and TRP623 of STAT-3 formed strong interactions with genipin. To further confirm whether genipin can directly bind to the STAT-3-SH2 domain, GST-tagged STAT-3-SH2 domain (42 KD; see below) was purified from *E. coli* (Fig. 2b). Then, SPR assay was performed to determine the binding affinity between genipin and STAT-3-SH2. SPR analysis results indicated that STAT-3-SH2 bound to genipin with a relatively low dissociation constant (KD) value (KD = 2.3 μM) (Fig. 2c). The activation of STAT-3 required phosphorylation on tyrosine and forming a dimer via phosphotyrosine/SH2 domain interaction [26]. Our results showed that genipin distinctly suppressed the interaction between purified STAT-3-SH2 and STAT-3 by GST pull-down assay (Fig. 2d). Next, FLAG-tagged and HA-tagged STAT-3 vectors were constructed and transfected into MHCC97L cells for validating whether genipin inhibits the dimerization of STAT-3. Our results suggested that HA-STAT-3 co-immunoprecipitated with FLAG-STAT-3 in MHCC97L cells and genipin blocked the interplay dose-dependently (Fig. 2e). In addition, genipin also inhibited STAT-1:STAT-3 heterodimer formation (Supplementary Fig. 2a). These results indicated that genipin might directly bind to the STAT-3-SH2 domain and inhibit the dimerization of STAT-3 or STAT-1:STAT-3. EGFR can also bind to the STAT-3-SH2 domain and activate STAT-3 [27]. GST pull-down results indicated that purified STAT-3-SH2 interplayed with EGFR and genipin exposure (20 μM) suppressed the complex formation (Fig. 2f). Then, whether genipin could induce the dissociation of the EGFR-STAT-3 complex was further explored. It was found that treatment with EGF can increase the binding ability of STAT-3 to EGFR in HCC cells, while treatment with genipin significantly suppressed these interactions (Fig. 2g). These results demonstrated that genipin directly bonded with the STAT-3-SH2 domain.

**Fig. 2:** Genipin directly binds with STAT-3-SH2 domain. (**a**) 3D docking results indicated that genipin could bind to SH2 domain in STAT-3. (**b**) Purified GST-tagged STAT-3-SH2 protein was analyzed by SDS-PAGE. Coomassie blue was used to stain the target protein. (**c**) Fitted curve for different concentrations of genipin binding to immobilized STAT-3-SH2 by “Affinity” model in the Biocore T300 evaluation software. Differently colored dots represent different concentrations of genipin. (**d**) Genipin-suppressed SH2-SH2 interactions. Purified STAT-3-SH2 domain was incubated with MHCC97L cell lysates after mixing with different dosages of genipin for 1.5 h and analyzed by GST pull-down assay. (**e**) Genipin suppressed the dimerization of STAT-3. MHCC97L cells transfected with HA and FLAG-tagged STAT-3 vectors were pre-treated with genipin, the interaction of FLAG-STAT-3 and HA-STAT-3 were validated by immunoprecipitation assay. (**f**) Purified STAT-3-SH2 domain was incubated with MHCC97L cell lysates after mixing with different dosages of genipin for 1.5 h; the interactions of STAT-3-SH2 with EGFR were validated by GST pull-down. (**g**) HCC cells (MHCC97L and HepG2) were pre-treated with different dosages of genipin and incubated with EGF; the interactions of STAT-3 with EGFR were validated by co-immunoprecipitation

### Genipin inhibits HCC cell proliferation and angiogenesis in vitro

The above results clearly demonstrated that genipin can inhibit STAT-3 activation. To evaluate the anti-cancer effect of genipin, its potential suppressive effect on HCC cell proliferation was examined by MTS assay. To our surprise, genipin remarkably inhibited HepG2 and MHCC97L cell viability dose-dependently. However, no significant inhibition effect on normal liver cells (LO2) was observed in our study (Fig. 3a). Western blotting results showed that the phospho-STAT-3 (Tyr-705) level was decreased after genipin treatment in HCC cells, but remained unchanged in normal liver cells (LO2) (Supplementary Fig. 3a). Next, whether STAT-3 inhibition is related to impaired cancer cell proliferation was further explored. STAT-3 vectors were transfected into MHCC97L cells, and over-expression of STAT-3 obviously reversed genipin-mediated tumor growth inhibition and STAT-3 target gene suppression (Fig. 3b). Furthermore, genipin (10 μM) could induce apoptotic cell death in HCC cells as indicated by western blotting and Annexin V/7AAD assay (Fig. 3c). Then, whether genipin inhibited colony formation in MHCC97L and HepG2 cells was further determined. As shown in Fig. 3d, genipin suppressed colony formation in MHCC97L and HepG2 cells in a dose-dependent manner. Accumulating evidence suggests that STAT-3 plays a critical role in angiogenesis under both pathological and physiological conditions, in addition to cell proliferation and survival [28]. It has been widely recognized that angiogenesis plays a pivotal role in cancer development, as malignant tumors need sufficient blood provision if the tumor is to grow beyond a few cubic millimeters in volume [29]. One of the most widely applied in vitro experiments to model the reorganization stage of angiogenesis is the tube construction assay. In our study, genipin failed to affect HUVEC viability (Supplementary Fig. 4a) or capillary-like structure construction (Supplementary Fig. 4b) in the culture medium. However, less well-formed capillary-like structures were built for HUVECs in the MHCC97L-conditioned medium after genipin (10 and 20 μM) treatment (Fig. 3e). In conclusion, the above results revealed that genipin might inhibit HCC proliferation and angiogenesis.

**Fig. 3:** Genipin inhibits HCC cell proliferation and angiogenesis. (**a**) MHCC97L, HepG2, or normal haptic cells (LO2) were treated with different dosages of genipin for 24 h. Cell viability was detected by MTS assay. (**b**) STAT-3 vector was transfected into MHCC97L cells. Cell viability was detected by MTS assay, and protein expression of STAT-3 target genes was examined by western blotting. (**c**) HCC cells were pre-treated with different concentrations of genipin for 24 h; cell apoptosis was analyzed by flow cytometry using Annexin V/7AAD commercial kit. Expressions of PARP and cleaved PARP were examined by western blot assay. (**d**) Colony formation assays were used to detect HCC cell proliferation ability. MHCC97L and HepG2 cells were incubated with 20-μM genipin for 2 weeks. Results were shown in the histogram from three independent experiments. (**e**) Angiogenesis was detected by tube formation assay. 1 × 10^5^ HUVECs were cultured on Matrigel. Cells were incubated with genipin for 10 h; representative images of tube formation were observed under an inverted microscope (Leica, Germany) and the relative tube numbers were analyzed. The data presented as mean ± SD. *P < 0.05 and **P < 0.01

### Genipin suppresses HCC cell invasion and reverses EMT process

The spread and metastasis of cancer cells may occur by invading the surrounding tissues and intravasating into blood or lymphatic circulation through the endothelium [30]. Herein, cell invasion ability was analyzed by Transwell assay using MHCC97L and HepG2 cells. Our results showed that genipin (10 μM) inhibited HCC cell invasion dose-dependently (Fig. 4a). Cancer invasion requires an extracellular matrix (ECM) and basement membrane degradation. Thus, fluorescent-gelatin degradation assay was applied to examine whether genipin suppresses ECM degradation by HCC cells. Our results suggested that MHCC97L cells significantly promoted ECM degradation in the control group, while genipin (20 and 50 μM) treatment reversed ECM degradation by HCC cells (Fig. 4b). 3D culture is an artificially created environment that provides functional and structural aspects of cancer development. In this study, our 3D culture results showed that genipin (20 and 50 μM) remarkably suppressed HCC cell invasion via the surrounding Matrigel (Fig. 4c). Epithelial-mesenchymal transition (EMT) is a key process in cancer metastasis by which epithelial cells lose their polarity and cell-cell adhesion and obtain invasive and migratory properties. During the EMT process, the expression of several epithelial and mesenchymal biomarkers significantly changed. Interestingly, genipin treatment notably decreased the expression of vimentin, fibronectin, and N-cadherin while increasing the expression of E-cadherin in HCC cells (Fig. 4d).

**Fig. 4:** Genipin suppresses HCC cell invasion and reverses EMT process. (**a**) MHCC97L and HepG2 cells were cultured in trans-well inserts (upper chamber). Images were obtained via optical microscope after genipin treatment 12 h later; invaded cells were calculated by three individual researchers. Scale bar 50 μm. (**b**) MHCC97L cells were cultured in FITC-conjugated gelatin (green) for 24 h. Phalloidin was applied to stain F-actin (red) and DAPI used to indicate nuclei (blue). Black area underneath the cell indicates gelatin degradation area; scale bar 20 μm. (**c**) To construct the 3D culture system, MHCC97L cells were seeded into a layer of Matrigel. Then, different dosages of genipin with DMEM and 15% Matrigel were added. Upper mixture was replaced every 24 h. Arrows indicate tubular structure formation on Matrigel. Images were obtained via optical microscope after genipin treatment 96 h later; scale bar 50 μm. (**d**) Protein expressions of vimentin, fibronectin, N-cadherin, and E-cadherin were validated by western blot and immunofluorescence staining (green). Nuclei were stained by DAPI (blue). Scale bar 20 μm. Data presented as mean ± SD. *P < 0.05, **P < 0.01, and ***P < 0.001

### Genipin suppresses cancer progression in HCC xenograft tumor models

To further explore whether genipin suppresses HCC progression in vivo, orthotopic mice xenograft models with MHCC97L cells were established. Then, DMSO (0.1%) (vehicle) or genipin was administrated daily by intraperitoneal injection. Figure 5a shows that genipin treatment (25 and 50 mg/kg) notably decreased tumor weight, which indicated that genipin could inhibit HCC progression in vivo. In addition, genipin treatment also significantly decreased the number of metastasis nodules in the lungs (Figs. 5b and c). Further studies demonstrated that genipin suppressed the protein expression of phospho-STAT-3 (Y705) and inhibited the expressions of STAT-3 target genes in primary liver tumor tissues (Figs. 5d and e). Furthermore, decreased vascular density was detected by CD31 staining in HCC tissues in genipin-treated mice (Fig. 5e). The survival rate of mice was analyzed to evaluate whether the metastasis inhibition effects of genipin could improve the overall survival rate. Our results showed that genipin significantly improved the survival rate of tumor-bearing mice. No mice in the vehicle group (*n* = 8) survived by day 40, whereas six mice survived by days 40 and 50 after genipin (50 mg/kg) treatment (Fig. 5f). In conclusion, the above results suggested that genipin could inhibit HCC metastasis and improve the overall survival rate in orthotopic transplantation HCC mice models.

**Fig. 5:** Genipin suppresses HCC progression and improves survival rate of tumor-bearing mice. MHCC97L cells (5 × 10^5^) were used to established orthotopic mice xenograft models. Tumor-bearing mice were administrated with DSMO or genipin by intraperitoneal injection (*n* = 8). (**a**) Tumor weight of primary liver cancer in mice was detected after DSMO (0.1%) or genipin treatment. (**b**) To evaluate lung metastasis in orthotopic transplantation HCC mice, lung tissues were dissected after DSMO or genipin treatment. Representative paraffin sections of lung tissue were stained with hematoxylin and eosin at 20× magnification. Scale bar 100 μm. (**c**) Lung metastasis was examined under anatomic microscope and number of metastasis nodules was calculated by three individual researchers. (**d**) Protein expression of p-STAT-3 (Y705) and target gene expression in primary liver tumors were detected by western blot assay. (**e**) Protein expressions of CD31 and phospho-STAT-3 were evaluated by immunohistochemical method. Scale bar 40 μm. (**f**) Overall survival was analyzed after DSMO or genipin treatment (0–50 d) in tumor-bearing mice. Genipin vs vehicle (25 mg/kg), *P* = 0.0002; genipin vs vehicle (50 mg/kg), *P* < 0.0001. Data presented as mean ± SD. **P < 0.01 and ***P < 0.001

### Anti-HCC effect of genipin in patient-derived HCC xenograft mice model

A patient-derived xenograft (PDX) mice model may retain more similarities to human cancers compared to a normal cell-line xenograft mice model. Previous studies have shown that PDX mice models may be useful for screening novel anti-cancer agents [31]. Herein, seven human surgical HCC tissue samples along with the peripheral normal liver tissues were collected from primary HCC patients (Supplementary Table 1). First, the protein expressions of STAT-3 and p-STAT-3 (Y705) in these surgical samples were detected. Our results indicated that the expressions of STAT-3 and p-STAT-3 (Y705) were notably reduced in HCC peripheral normal liver tissues compared to tumor tissues (Fig. 6a). These results suggested that the activation of STAT-3 is up-regulated in tumor cells derived from HCC patients. After establishing the PDX mice model, the protein expressions of STAT-3 and p-STAT-3 (Y705) in tumor-bearing mice were examined. No obvious changes were found in the expression of p-STAT-3 (Y705) in F0, F1, F2, and F3 passages (Fig. 6b). The above results indicated that the activity of STAT-3 was not changed in patient-derived HCC xenograft mice after serial passages culture. The F3 passages mice were divided into DMSO (0.1%) and genipin (25, 50 mg/kg/d) treatment groups (*n* = 8). After genipin treatment, the HCC growth in mice was significantly suppressed (Fig. 6c). The tumor volume in the genipin treatment (25 and 50 mg/kg/d) group was 597.43 and 401.26 mm^3^, respectively. In contrast, the tumor volume in the vehicle treatment group was 1452.24 mm^3^ (Fig. 6d). In addition, the tumor weight in the liver remarkably decreased after genipin (25 and 50 mg/kg/d) treatment (Fig. 6e). Interestingly, genipin also decreased the protein levels of p-STAT-3 (Y705) and STAT-3 target genes (Bcl-2, VEGF, and Survivin) in the mice model (Fig. 6f). Immunohistochemistry assay further confirmed the decreased expression of p-STAT-3 (Y705) as well as the tumor vascular density (CD 31+) in HCC samples from PDX mice after administration with genipin (25 and 50 mg/kg/d) (Fig. 6g).

**Fig. 6:** Genipin exhibits anti-HCC effects in PDX mice model. (**a**) Protein expression of STAT-3 and p-STAT-3 (Y705) in human HCC tissue and para-carcinoma tissue were examined by western blot assay. (**b**) Graphical representation of constructing PDX mice model. Protein expression of STAT-3 and p-STAT-3 (Y705) were detected in F1, F2, and F3 generation. (**c**) Tumor sizes were measured after genipin treatment in PDX model (*n* = 8). (**d**) Tumor volume in PDX mice was examined after genipin treatment (*n* = 8). (**e**) Tumor weight in PDX mice was examined after genipin treatment (*n* = 8). (**f**) Expression of p-STAT-3, STAT-3, Survivin, Bcl-2, and VEGF was examined by western blotting in HCC tissues. (**g**) Expression of CD31 and p-STAT-3 was validated by immunohistochemistry assay in HCC tissues. Scale bar 40 μm. Data presented as mean ± SD. **P < 0.01 and ***P < 0.001

### Genipin inhibits proliferation of other cancer cells

Considering that STAT-3 signaling regulates oncogenic pathways in various tumor cells, it was hypothesized that genipin might also inhibit the growth of other cancer cells. Figure 7a shows that genipin (20 and 50 μM) exposure resulted in the growth inhibition of various kinds of cancer cells. In addition, genipin notably suppressed the STAT-3 signal pathway in these tumor cells. Figure 7b shows that the activation of p-STAT-3(Y705) was significantly inhibited by genipin treatment in various non-HCC cancers.

**Fig. 7:** Genipin suppresses proliferation of various non-HCC cancer cells. (**a**) Colon, gastric, ovarian, breast, prostate, cervix, and pancreas cancer cells were pretreated with genipin (20 and 50 μM). Living cells were detected by MTS assay after 36 h of incubation. (**b**) Various non-HCC cancer cells were pre-treated with genipin (20 and 50 μM) for 12 h. Expressions of p-STAT-3 and total STAT-3 were examined by western blot assay. Data presented as mean ± SD. **P < 0.01 and ***P < 0.001

### Potential toxicity of genipin on tumor-bearing mice

To evaluate the potential toxicity of genipin in vivo, the effects of genipin on kidney and liver functions in tumor-bearing mice were further examined. No obvious changes in serum creatinine, blood urea nitrogen, aspartate transaminase (AST), and alanine transaminase (ALT) levels between genipin and DMSO group were detected (*p* > 0.05) (Supplementary Table 2). In addition, body-weight changes in mice were detected every 7 d. No significant loss of body weight was detected after genipin treatment (Supplementary Fig. 5a). Furthermore, H&E staining results indicated no obvious histological changes between genipin-treated mice and control mice (Supplementary Fig. 5b). In conclusion, these data suggested that genipin exhibits no significant adverse effects on mice at the therapeutic dosage.

## Discussion

Discovering novel agents from natural products for HCC treatment may provide promising therapeutic drugs for improving patient survival [32, 33]. In the current study, it was found that a small natural compound, genipin, could inhibit STAT-3 activity in vitro and in vivo. Our molecular docking study indicated that genipin could bind to the SH2-STAT-3 domain, which was further confirmed by in vitro studies. For the first time, to the best of our knowledge, it was demonstrated that genipin could inhibit HCC progression by targeting the STAT-3 signal pathway (Fig. 8).

**Fig. 8:** Graphic illustration of signaling underlying molecular mechanism of anti-HCC effects of genipin

Previous studies have shown that genipin could induce apoptosis in HCC cells, detected by caspase activation, cytochrome C release, and changes in cellular morphology [34]. Further studies indicated that genipin-mediated HCC apoptosis might induce by NADPH oxidase-dependent generation of ROS, which resulted in JNK activation. Another study by Wang et al. showed that genipin might inhibit the intrahepatic metastasis with few adverse effects, and p38/TIMP-1/MMP-2 signaling may be involved as the key mechanism of genipin’s anti-metastasis effects [35]. Another recent study found that 50-mM genipin decreased the migratory distance by 43 and 72% in HCC cell lines. Genipin might down-regulate matrix metalloproteinases genes and protein expressions; decrease the expression of nuclear factor kappa-light-chain-enhancer of activated B cells, phosphorylated protein kinase B, urokinase-type plasminogen activator, phosphorylated mitogen-activated protein kinase, and activator protein 1; and up-regulate tissue inhibitor metalloproteinases genes as well as the protein expression in HCC [36]. Aside from its potential anti-HCC effects, genipin also showed therapeutic potential in hepatitis, hepatic injury, non-alcoholic fatty liver disease, and other non-cancer hepatic diseases, which might prevent the tumorigenesis of HCC [37]. Although genipin has shown inhibitory potency in HCC cells, its effects on STAT-3 activity in HCC has not been reported yet. Herein, for the first time, the anti-HCC effects of genipin and the involvement of STAT-3 in these effects were explored.

The SH2 domain is a structurally conserved protein domain contained within the STAT-3 protein. SH2 domains can promote STAT-3 dimerization by docking to phosphorylated tyrosine residues on STAT-3 [38]. This dimerization changes the STAT-3 conformation and facilitates target DNA recognition as well as regulation of gene expression. Our in silico studies suggested that genipin could bind to the SH2-STAT-3 domain, which was further confirmed by SPR study. In addition, co-immunoprecipitation assay indicated that genipin inhibited STAT-1:STAT-3 heterodimerization and STAT-3:STAT-3 homodimerization. In previous research, Mahalapbutr et al. found that the SH2 domain was critical for EGFR and STAT-3 interaction and subsequent STAT-3:STAT-3 homodimerization [39]. In our study, it was revealed that genipin could suppress EGFR-STAT-3 interaction and further inhibit STAT-3 dimerization. The STAT-3 protein has two critical phosphorylation sites, Ser727 and Tyr705, for its activation. However, genipin failed to phosphorylate STAT-3 on the Ser727 site in this study. Thus, it is speculated that genipin can inhibit STAT-3 activity by suppressing STAT-3 phosphorylation on the Tyr-705 site.

In this study, genipin suppressed HCC cell proliferation by regulating the expression of survivin, Mcl-1, and Bcl-2 genes. However, genipin failed to affect several common signal pathways that have a close association with cancer proliferation, e.g., the mTOR, STAT-5, STAT-1, STAT-2, and MAPK pathways. Thus, it is speculated that genipin might inhibit HCC cell proliferation by specifically suppressing STAT-3 activity. Ulaganathan et al. revealed that STAT-3 was constitutively activated in malignancy instead of normal tissues [40, 41]. Interestingly, our results showed that genipin selectively suppressed HCC cell proliferation without significant toxicity in normal cells. These findings suggested that STAT-3 might be a promising therapeutic target for cancer treatment with few side effects. The vascular endothelial growth factor (VEGF), originally known as the vascular permeability factor (VPF), is a signal protein that can stimulate the formation of blood vessels in cancer development [42]. Sim et al. showed that STAT-3 could regulate the expression of VEGF in various types of cancers [43]. Herein, our results demonstrated that genipin remarkably decreased the expression of VEGF in HCC cells. Chromatin immunoprecipitation results confirmed that STAT-3 could regulate the expression of VEGF and inhibit STAT-3 binding to the promoter region of VEGF. In addition, HUVEC tube construction assay showed that less well-formed capillary-like structures were built for HUVECs in the tumor-conditioned medium derived from genipin-treated cells. In vivo studies further confirmed the decreased cancer vascular density in mice after genipin treatment by IHC assay. In conclusion, the decreased expression of VEGF regulated by STAT-3 might contribute to genipin-induced cancer angiogenesis suppression. One insufficiency of the present study is that Akt pathway in genipin-induced HCC proliferation inhibition was not investigated. Previous studies showed that regulation in the Akt pathway could affect growth factors, receptor tyrosine kinases, Ras, and the PI3K p110 sub-unit, resulting in abnormal cancer cell proliferation [30, 44]. Therefore, in future studies, further exploration of the potential role of the Akt pathway in genipin-induced HCC suppression is planned.

Cancer metastasis is a pathological process in which malignant cells spread from a primary site to a different site within the host’s body [45, 46]. The degradation of ECM plays a pivotal role in the process of metastasis. MMP-2, a type IV collagenase, can facilitate ECM degradation and promote cancer metastasis. Previous studies showed that STAT-3 could regulate the expression of MMP-2 in cancer cells [47]. In our study, genipin notably suppressed the expression of MMP-2 in HCC cells and inhibited the degradation of ECM. The epithelial-mesenchymal transition (EMT) is a process by which epithelial cells lose polarity and adhesion ability, which can promote cancer cell metastasis [48]. Xiong et al. found that STAT-3 might directly induce EMT progression and modulate ZEB1 expression in colon cancer cells. Knockdown of STAT-3 can up-regulate the expressions of E-cadherin and down-regulate N-cadherin and vimentin in colon cancer [1]. According to our results, genipin can also regulate EMT-relevant protein expression in HCC. Furthermore, genipin treatment remarkably suppressed HCC lung metastasis in a xenograft mice model. The above results suggested that genipin might inhibit MMP-2 expression and block the process of EMT in HCC by targeting STAT-3 activity, which could suppress HCC metastasis.

A patient-derived xenograft (PDX) mice model refers to the transferring of human cancer samples to immunodeficient mice after surgical operation. As PDX can be passaged without in vitro processing procedures, a PDX model enables the propagation and expansion of human cancers without oblivious genetic transformation of cancer cells over multiple murine generations [49]. Within a PDX model, human cancer can grow in a physiologically relevant cancer microenvironment that mimics the hormone, nutrient, and oxygen levels that are observed in primary human cancer tissues [50]. Thus, a PDX model shows significant advantages over established cancer cell lines in cancer research. Herein, it was found that genipin exhibits notable therapeutic effects in an HCC PDX mice model. Our in vivo results indicated that the expression level of p-STAT-3 (Y705) was higher in cancer tissues than para-carcinoma tissues. Furthermore, HCC PDX mice still exhibit a high expression of p-STAT-3 (Y705) after continuous passage.

In conclusion, genipin showed therapeutic potential for HCC treatment by directly interacting with the SH2-STAT-3 domain, which suppressed the activity of STAT-3. Our study may form the baseline research for future clinical trials and suggests genipin as a novel inhibitor of STAT-3. In addition, more in-depth research could be conducted to explore the potential role of genipin in combination with chemotherapy for HCC in future studies.

## Conclusions

In conclusion, in this study, genipin showed therapeutic potential for HCC treatment by interacting with the SH2-STAT-3 domain and suppressing the activity of STAT-3. In the future, further research is planned to explore the potential role of genipin in combination with chemotherapy or radiotherapy for HCC treatment.

## Supplementary information

**Additional file 1: Supplementary Figure 1.** Genipin failed to affect the expression of PTPases or activation of STAT-1, STAT-2, STAT-5, mTOR and MAPK signal pathways. (a) For validating the effects of genipin on the expression of PTPases , western blot assay was applied after genipin treatment.(b) For validating the effects of genipin on the activation of STAT-5, STAT-2, STAT-1, western blot assay was applied after genipin treatment. (c) For validating the effects of genipin on the activation of MAPK and mTOR signaling pathways, western blot assay was applied after genipin treatment. **Supplementary Figure 2.** Genipin inhibits the formation of STAT3-STAT1 heterodimer. (a) MHCC97L cells were transfected with HA-tagged STAT1 and FLAG-tagged STAT3 and pretreated with genipin, the binding ability of STAT3-STAT1 was validated by western blotting and immunoprecipitation assays. **Supplementary Figure 3.** Genipin suppresses the protein expression of p-STAT3 (Y705) in HCC cells. (a) HCC and normal liver cells were treated with genipin for 12 h, cells extracts were prepared and protein expressions were examined by western blot assay. **Supplementary Figure 4.** Genipin failed to affect the proliferation of HUVECs and capillary structure formation. (a) HUVECs were treated with genipin (5,10, 20, 50 μM ) for 24 h and examined by MTS assay. (b) 5×10^3^ HUVECs were cultured in 24-well plates, then, genipin (10, 20, 50 μM ) were exposed to cells.. After 12 h incubation, Tubular structures were observed by inverted microscope(Carl Zeiss Vision, Germeny) and analyzed by Pro-Image ( Media Cybernetics, USA) software. The data represents mean ± SD. Scale bar = 20 μm. **Supplementary Figure 5.** The potential cytotoxicity of genipin *in vivo*. (a) Nude mice were administrated with genipin (50 mg/kg/day) or DMSO by i.p. injection for 4 weeks (*n* = 6). The body weight was detected each week. (b) H&E staining results of brain, heart, lung, kidney and spleen organs from DMSO group and genipin group. Scale bar=20 μm. **Supplementary Table 1**. The information of HCC patients with tumor resection operation **Supplementary Table 2.** The effects of genipin on kidney and liver functions in nude mice **Supplementary Table 3.** The primer sequences used in RT-PCR assay

## Data Availability

All the data and materials supporting the conclusions were included in the main paper.

## Abbreviations

PDX: Patient-derived xenograft
DMSO: Dimethylsulfoxide
HCC: Hepatocellular Carcinoma
STAT-3: Signal Transducers and Activators of Transcription-3
MMP-2: Matrixmetallo proteinase-2
EMT: Epithelial-mesenchymal transition
VEGF: Vascular endothelial growth factor
VPF: Originally known as vascular permeability factor
ECM: Extracellular matrix
SPR: Surface plasmon resonance
PTPases: Protein tyrosine phosphatases
